# Genetic variation and relationships in the mitochondrial DNA D-loop region of Qinghai indigenous and commercial pig breeds

**DOI:** 10.1186/s11658-018-0097-x

**Published:** 2018-07-03

**Authors:** Junxia Zhang, Baochun Yang, Xiaocheng Wen, Guoqiang Sun

**Affiliations:** 1 State Key Laboratory of Plateau Ecology and Agriculture, Qinghai University, Xining, 810016 Qinghai China; 2 College of Agriculture and Animal Husbandry, Qinghai University, Xining, Qinghai China

**Keywords:** Mitochondrial DNA, Genetic variation, Bamei pig, Commercial pig

## Abstract

**Background:**

Bamei pigs are special germplasm resources in Qinghai. In the specific environment of the Qinghai plateau, local breeds, through long-term natural and artificial selection, have acquired a relatively stable population structure and genetic diversity. This study revealed Bamei pigs’ genetic diversity at the molecular level and the degree of introgression of commercial breeds into Bamei pigs.

**Methods:**

The mitochondrial DNA D-loop region was amplified and sequenced using the ABI 3130 DNA sequencer. Sequences were collected, edited and aligned using the MEGA 5.0, DNASTAR and ClustalX 1.81 software. Haplotypes of all sequences and genetic diversity were analyzed by DnaSP 5.0 software.

**Results and conclusions:**

We identified a total of 73 polymorphic sites in our 489 novel sequences, including 1 single variable site and 72 parsimony informative sites.

Genetic diversity was analyzed in this study. The results showed that haplotype diversity, nucleotide diversity and the average number of nucleotide differences of Bamei pigs were lower than those of commercial pigs. Synthetic evaluation of genetic diversity through principal component analysis indicated that Bamei pigs also showed low genetic diversity. In summary, the results of sequence analysis showed that Bamei pigs were low in genetic diversity, and the introgression of commercial pigs into Bamei pigs was serious.

## Background

With the high intensification of pig production, highly productive breeds became predominant in the pig production system, and the quantity of indigenous breeds was decreased, so breed resource protection become more important [1]. The Bamei pig is the indigenous pig breed in Qinghai Province of China, where there is a plateau continental climate. Under the influence of the ecological environment and natural and artificial selection, the Bamei pig was developed, which has the characteristics of good adaptability, high resistance, large litter size, good maternal qualities, high fat deposition ability, good meat quality and flavor, genetic stability, strong inbreeding resistance, adaptation to cold climate conditions and extensive feeding and management. However, they have some shortcomings, for example, slow growth, low lactation quantity, and low fattening benefit [2]. In the past 50 years, Qinghai Province has introduced some pig breeds such as Berkshire, white, Landrace, Duroc, Hampshire, England, Yorkshire and other foreign breeds, which were crossed with the Bamei pig through an economic hybrid and three-way hybrid. The offspring were fed with high nutritional diets. Although the production performance was increased, the Bamei pig breed is at risk of extinction [3].

mtDNA sequence analysis has enabled important investigation of the origin and diversification of animal populations [4–8]. mtDNA contains the displacement (D)-loop, containing regulatory sequences controlling both replication and transcription of mtDNA [1, 9]. In the present study, we examined sequence variation in mtDNA from Bamei pig populations and commercial pig populations. We also assessed the relative impact of commercial pigs on Bamei pig populations. This study aimed to acquire information on Bamei pig genetic diversity. The findings will be helpful for conservation and sustainable use of Bamei pig resources.

## Methods

### Sampling and sequencing

A total of 489 samples, including 489 individuals (4 pig breeds) distributed in Qinghai Province of China, were collected. (Information on collected samples is provided in Table 1.) Only ear tissues were collected into microcentrifuge tubes containing 75% ethanol, and preserved at − 80 °C. Animals were released immediately following treatment of the wounds with antiseptic.

**Table 1:** Characteristics of samples

Breed/population	Category	Sample size	Source	Sampling site
Bamei pig	Indigenous	115	Ear tissue	Qinghai Province
Duroc	Commercial	101	Ear tissue	Qinghai Province
Landrace	Commercial	108	Ear tissue	Qinghai Province
Yorkshire	Commercial	165	Ear tissue	Qinghai Province
Total		489		

Genomic DNA was extracted using the phenol-chloroform extraction method [10]. A fragment of the D-loop region was amplified using the primers 5′-CCAAAAACAAAGCAGAGTGTAC-3′ and 5′-CGTTATGAGCTACCGTTATA-3′. The PCR reaction mixture consisted of 25 μL, containing 12.5 μL 2 × *Eco Taq* PCR Supermix containing 1 U Taq polymerase, 500 mΜ dNTPs, and 10×Taq buffer (Beijing TransGen Biotech Co., Ltd., China), 0.1 μg of template DNA, 0.4 μL of 10 pmol/mL of each primer and 11.6 μL of ddH_2_O. The cycling conditions were initial denaturation at 94 °C for 5 min, followed by 33 cycles of 94 °C for 30 s, 56 °C for 30 s and 72 °C for 30 s, and a final extension for 5 min at 72 °C. Amplified DNA fragments were purified following agarose gel electrophoresis and sequenced using the ABI 3130 DNA sequencer (Applied Biosystems, Foster City, CA, USA).

### Data analysis

A total of 489 mtDNA D-loop sequences were obtained and analyzed in this study, including 115 sequences from indigenous pigs (Bamei pigs) and 374 sequences from commercial pigs (Duroc, Landrace and Yorkshire).

Original sequence data were obtained using the ABI PRISM DNA sequencer software. Sequences were edited using the DNASTAR software and aligned using ClustalX 1.81 [11]. In all sequences the length of alignment was reduced to 435 bp, and these were used to perform additional analyses. In addition, the haplotypes of all sequences and genetic diversity were analyzed using DnaSP 5.0 software [12]. Correlation analysis and principal component analysis (PCA) were investigated by SPSS 19.0.

## Results

### Genetic diversity analysis

The 435 bp control region of mtDNA was used to analyze single nucleotide polymorphisms (SNPs) for all 489 sequences. No insertion/deletions (indels) were detected in our novel sequences. We identified a total of 73 polymorphic sites, including 1 single variable site and 72 parsimony informative sites. The four types of nucleotide mutations identified were transitions, transversions, insertions and deletions. The transition: transversion ratio R (Ts/Tv) was 13.29:1, indicating a strong transitional bias that is common in mammalian mitochondrial evolution [13].

The genetic diversity of Bamei pigs and commercial pigs was calculated (Table 2). Haplotype diversity (Hd) of pig populations was between 0.491 and 0.856. All commercial pigs had high haplotype diversities of over 0.7. Yorkshire had the highest haplotype diversity (0.856 ± 0.018). Bamei pigs had the lowest haplotype diversity (0.491 ± 0.055). The result showed that haplotype diversity of Bamei pigs was lower than that of commercial pigs. Nucleotide diversities (Pis) were in the range 0.00264–0.01559. Landrace had the highest nucleotide diversity (0.01564), while Bamei pigs had the lowest (0.00264). Average nucleotide diversity of commercial pigs was higher than that of Bamei pigs. For all varieties of pigs the average number of nucleotide differences (Ks) was between 6.815 and 1.15; for Landrace it was the highest (6.815), and for Bamei pigs the lowest (1.15) – lower than for all commercial pigs.

**Table 2:** Parameters for determination of genetic diversity of pig populations

Code	Breed/Population	Size	S	H	Hd ± SD	Pi	K
CHN-QH	Bamei	115	10	10	0.491 ± 0.055	0.00264	1.15
DUR	Duroc	101	18	11	0.732 ± 0.033	0.00947	4.12
LAN	Landrace	108	18	18	0.853 ± 0.02	0.01567	6.815
YOR	Yorkshire	165	27	24	0.856 ± 0.018	0.01559	6.768

S: Number of polymorphic (segregating) sites

H: Number of haplotype

Pi: Nucleotide diversity, Nei 1987, eqs. 10.5 or 10.6 (Masatoshi Nei)

K: Average number of nucleotide differences; Tajima 1983, eq. A3 (Tajima)

Hd ± SD: Haplotype (gene) diversity and sampling variance, Nei 1987, eqs. 8.4 and 8.12 but replacing 2n with n. The standard deviation (or standard error) is the square root of the variance (Masatoshi Nei) [13]

The correlation of Pi, Hd and K was analyzed using SPSS 19.0 (Table 3). The results showed that Hd, Pi and K were positively correlated with each other, which indicated that all three indexes influenced the abundant degree of genetic diversity. Principal component analysis (PCA) was used for synthetic assessment of genetic diversity. The results are shown in Table 4. We obtained a synthesized assessment score (Fz). The Fz score indicated the highest genetic diversity in Landrace and the lowest for Bamei pigs.

**Table 3:** Correlation matrix between indexes

Item	Hd	Pi	K
Hd	1.000	.990	.990
Pi	.990	1.000	1.000
K	.990	1.000	1.000

**Table 4:** Rank and general scores of principal components of different populations

Code	Breed/population	F_Z_ (F_1_)	Rank
CHN-QH	Bamei	−2.345	4
DUR	Duroc	−0.132	3
LAN	Landrace	0.405	1
YOR	Yorkshire	0.001	2

### Haplotype analysis of sequences

The 435 bp control region of mtDNA was used to calculate haplotypes for all 489 sequences. In total, 43 haplotypes were identified according to the distribution of variable sites (Table 5). Distribution frequencies of haplotypes indicated no equilibrium. The highest frequency haplotype was Hap34, which was shared by 97 sequences. The lowest frequency haplotypes were 26, and each haplotype harbored a sequence. Another 17 haplotypes were shared by two or more sequences. Hap31 and Hap34 were advantageous haplotypes which were present in more than 90 sequences. The Bamei porcine population shared 11 haplotypes. The commercial porcine population shared 36 haplotypes.

**Table 5:** The distribution of variable sites of mtDNA D-loop in pig populations

H	Polymorphism sites 22456771111111111111111222222222222223333333333444 38322681122333445558888113344477788890001124699001 0115268464592356253612924703951270444012674	CHN-QH	DUR	LAN	YOR	Total
H1	CGAAT-CCGAAAA-TTTTGTTCTATAATCGTATCCAGCCTGATAGTCCTC				6	6
H2	.....-.T..TG.CACC.A....G....T.......A..C..C..C.T..			3	15	18
H3	T....-.T.TTG.CACC.A.........T.......A..C..C..C.T..		4			4
H4	.....A.T..TG-CACC.A.........T.......A.....C..C.T..				1	1
H5	.....-.T..TG.CACCCA.T....T..A..C..C..C.T..			1		1
H6	.....-.T..TG.CACC.AC........T...CT.GA..C..C..C.TC.		44	23	21	88
H7	.....-TTA..G.CACC.A.........T....T..A..C..CT.C.T..			2	1	3
H8	.....-.T...G.CACC.A..T......T.......A..C..C..C.T..			2	2	4
H9	.....-.T...G.-A.C..C........T.......A..C..C..C.T..			1		1
H10	.....-.......-A....C................A..C..C.......				2	2
H11	.....-.......-A....CC...............A..C..C..C.T..		1		3	4
H12	.....-.......-A....C........T..........C..C..C.T..		3	12	6	21
H13	....C-.......AA..................T.....C..C..C.T..			8	2	10
H14	....C-.......A-.................CT............TT..			2		2
H15	.....-.......CA.C.............T.............T..				1	1
H16	.....-.......-A....C.............T..........A..T..			1	1	2
H17	.....-.......-A....C.........A.G...............T..		27	1	13	41
H18	.....-.......-A....C.........A...T.............T..				1	1
H19	.....-.......-A....C.....................G.....T..		1			1
H20	.....-.......-A....C................A..........T..				1	1
H21	.....-.......-A....C................A.............			2	2	4
H22	.....-.......-A....C........T....T...........C.T..				1	1
H23	.....-.......CA.C........T....T.............T..		7		3	10
H24	.....-.......-A....C........T....TT............T..				2	2
H25	.....-.......-A....C......G.T....T..A..........T..		1	8		9
H26	.....-.......-A....C........T....T.............T.T			1		1
H27	.....-.......-A....C........T...........A......T..		1			1
H28	.....-.......-A....C........T.G..T......A......T..	1				1
H29	.AG..-.T..TG.CACC.A.........T.......A..C..C..C.T..	1				1
H30	.....-.T..TG.CACC.A.........T.......AT.C..C..C.T..		1			1
H31	.....-.T..TG.CACC.A.....C...T.......A..C..C..C.T..	10	6	29	51	96
H32	.....-.T..TG.CACC.AC........T.......A..C.....C.T..		1			1
H33	.....-.T..TG.CACC.A.........T..........C..C..C.T..	6				6
H34	.....-.T...G.CACC.A.....CG..T.......A..C.....C.T..	81		4	12	97
H35	...G.-.T..TG.CACC.A.........T.......A..C..C..C.T..	1				1
H36	.....-.T..TG.CACC.A.........T.......A..C..C..C....	4		2	3	9
H37	.....-.T..TG.CACC.A........CT.......A..C..C..C.T..	8				8
H38	.....A.T..TG.CACC.A.........T.......A..C..C..C.T..	1				1
H39	.....-.T..TG.CACC.AC........T....T.GA..C..C..C.T..	1				1
H40	....C-.......AA.................CT............TT..				1	1
H41	.....-.......-A....C........T.........T........T..	1	4	5	11	21
42	.....-.......CA....C..............................				1	1
H43	.....-.......-A...................................			1	2	3

H1–43: Different haplotypy

CHN-QH: Bamei pig population

DUR: Duroc pig population

LAN: Landrace pig population

YOR: Yorkshire pig population

### Introgression of commercial pigs into Qinghai indigenous pigs

Forty-three haplotypes in 489 individuals from indigenous and commercial breeds were identified. Eleven haplotypes were identified in indigenous pigs and 36 haplotypes were identified in commercial pigs. Seventeen shared haplotypes were identified and distributed in 96 indigenous and 123 commercial pigs. The ratio of the number of indigenous pigs with shared haplotypes and the total of indigenous pigs (Sc/S) showed the degree to which indigenous pigs were affected by commercial pigs. Sc/S was 83.48% (Table 6). Our data showed that Bamei breed was impacted by commercial breeds (Landrace, Yorkshire and Duroc).

**Table 6:** Analysis of native pig haplotypes shared with commercial pigs

Code	Breed	Sc	S	Sc/S
CHN-QH	Bamei	96	115	83.48%

## Discussion

### Genetic diversity of Bamei and commercial porcine populations

Hd, Pi and K were the basic parameters which were used to assess genetic diversity. Hd is a measure of the uniqueness of a particular haplotype in a given population [14], which reflects haplotype abundance in a population. Pi and K measure the degree of intrapopulation haplotype mutation [11]. Our study examined genetic diversity of Bamei and commercial porcine populations, and the results showed that the genetic diversities of both Bamei and commercial porcine populations were low, which is consistent with the trend of the genetic diversity of global livestock populations declining [15]. Bamei pigs had the lowest haplotype diversity due to commercial hybridization. Bamei pigs have a low growth rate, so commercial pigs were used to cross with Bamei pigs to improve their performance. The Bamei population is, therefore, becoming smaller, and it is even becoming a critically endangered breed. Principal component analysis (PCA) is a statistical procedure to reduce the dimensionality of a data set by transformation to a new set of variables (the principal components) to summarize the features of the data [16]. The diversity parameters, including Hd, Pi and K, were analyzed using PCA. Fz ranged from − 2.345 to 0.405, and its rank indicated that Bamei pigs had the lowest level of diversity, while Landrace had the highest diversity. This is consistent with the analysis of other studies which showed that indigenous pigs have a lower level of genetic diversity [17–19]. Genetic diversity is essential for continued breeding. This is especially true in the situation where future breeding goals differ from current goals [20]. The Bamei pig as an indigenous porcine breed could be a useful resource for porcine production, so the protection of the Bamei pig from extinction will be important.

### Introgression of commercial breeds into Qinghai indigenous breeds

Chinese indigenous breeds are known for their low growth rate and poor feed conversion efficiency, while commercial breeds are characterized by high meat yield, fast growth rate and excellent feed efficiency, so commercial breeds have been extensively applied in the swine industry [21]. Increasing use of commercial lines threatens indigenous breeds and decreases genetic diversity. The Bamei pig similarly faces the threat of extinction due to the introgression of commercial pigs. Shared haplotypes were identified in 83.48% of Bamei pigs. Ninety-six haplotypes that were shared with commercial pigs were identified in 115 Bamei pigs. The reason for a high shared haplotype frequency in the Bamei population was crossbreeding with commercial lines. Current commercial lines were introduced and crossed with indigenous breeds, increasing the lineage of commercial lines. Despite its potentially economically unfavorable characteristics, the Bamei pig was recognized as an important genetic resource of the indigenous pig population due to specific traits (indigenous adaptation, strong adversity resistance, good maternal qualities). Additionally, the Bamei pig population was becoming small. The breeders are trying to maintain the Bamei pig breed and increase its number, so the founder effect might occur, which could result in a reduction in genetic diversity.

## Conclusions

Our results showed that diversity parameters, such as haplotype diversity, nucleotide diversity and the average number of nucleotide differences, of Bamei pigs were lower than those of commercial pigs. Synthetic evaluation of genetic diversity through principal component analysis indicated that Bamei pigs also have low genetic diversity. The introgression of commercial pigs into Bamei pigs was serious due to the influence of commercial pigs.
